# Efficacy and safety of nonsteroidal mineralocorticoid receptor antagonists for renal and cardiovascular outcomes in patients with chronic kidney disease: a meta-analysis of randomized clinical trials

**DOI:** 10.3389/fphar.2024.1338044

**Published:** 2024-02-27

**Authors:** Qianlan Chen, Guocui Wei, Yanping Wang, Xiuxia Li, Qian Zhao, Ling Zhu, Qing Xiao, Xuan Xiong

**Affiliations:** Department of Pharmacy, Sichuan Provincial People’s Hospital, School of Medicine, University of Electronic Science and Technology of China, Chengdu, China

**Keywords:** nonsteroidal mineralocorticoid antagonist, chronic kidney disease, cardiovascular events, randomized controlled trial, meta-analysis

## Abstract

**Objective:** To systematically review the efficacy and safety of nonsteroidal mineralocorticoid receptor antagonists (MRAs) in chronic kidney disease (CKD).

**Methods:** We systematically searched six databases to identify randomized controlled trials (RCTs) about nonsteroidal MRAs for CKD, from inception to 22 August 2023. Two reviewers independently screened the retrieved articles, extracted data, and assessed the risk of bias of included RCTs using the Cochrane risk of bias tool. We then conducted meta-analysis of the data using Stata 17.0 software.

**Results:** 11 RCTs (n = 15,817) were included in this meta-analysis. Compared with placebo, nonsteroidal MRAs significantly reduced the proportion of patients with ≥40% decline in estimated glomerular filtration rate (eGFR) from baseline [RR = 0.85, 95% CI (0.78, 0.92), *p < 0.001*], although the magnitude of eGFR reduction was greater [WMD = −2.83, 95% CI (−3.95, −1.72), *p < 0.001*]. The experimental group also had lower incidence of composite renal outcome [RR = 0.86, 95% CI (0.79, 0.93), *p < 0.001*] and greater reduction in urine albumin-to-creatinine ratio (UACR) from baseline [WMD = −0.41, 95% CI (−0.49, −0.32), *p < 0.001*], as well as reduced cardiovascular events [RR = 0.88, 95% CI (0.80, 0.95), *p* = 0.003]. MRAs did not increase any adverse events compared to placebo [RR = 1.00, 95% CI (0.99, 1.01), *p* = 0.909], but had higher incidence of hyperkalemia [RR = 2.05, 95% CI (1.85, 2.280), *p* < 0.001]. Compared with eplerenone, there was no significant difference in the proportion of patients with ≥40% decline in eGFR [RR = 0.57, 95% CI (0.18, 1.79), *p = 0.335*] or hyperkalemia [RR = 0.95, 95%CI (0.48, 1.88), *p* = 0.875].

**Conclusion:** Nonsteroidal MRAs can reduce the incidence of end-stage renal disease and cardiovascular adverse events in patients. Although there was still a risk of hyperkalemia compared to placebo, there was no significant difference in any adverse events compared to either placebo or eplerenone. It has become a new option for drug treatment of CKD patients, but more clinical trials are still needed to verify its efficacy and safety. Especially further direct comparison of the nonsteroidal MRAs to eplerenone in view of the relatively small number of patients reviewed are needed.

## 1 Introduction

The worldwide prevalence of chronic kidney disease (CKD) stands at 11.1%, with rates of 10.4% among men and 11.8% among women. This translates into an absolute global count of 843.6 million individuals living with CKD (Jager et al., 2019). The 2016 report of the China Kidney Disease Data Network (CK-NET) showed that patients with CKD constituted 4.86% of all admissions in tertiary hospitals in China (Zhang et al., 2020). CKD is one of the most prevalent chronic conditions, and its diagnosis and treatment outcomes significantly impact the final outcome. Regarding the etiology of CKD, the most commonly coded causes included diabetes (26.70%), hypertension nephropathy (HTN, 21.39%), obstructive nephropathy (ON, 16%), and glomerulonephritis (GN, 14.41%) (Zhang et al., 2020). Individuals with CKD are at an elevated risk of developing cardiovascular disease, which often clinically manifests as heart failure. Conversely, patients with heart failure commonly exhibit reduced kidney function. The connections between the kidneys and the cardiovascular system are gradually being unraveled (Haynes et al., 2020). In conclusion, it is imperative to discover medications that safeguard the heart and kidney functions, and mitigate the likelihood of terminal events.

A large number of mineralocorticoid receptors (MR), are distributed in the human body. Their physiological ligands are aldosterone and cortisol, and progesterone or androgens and their derivatives can also bind to MR (Rupprecht et al., 1993). Under various pathological conditions, the expression level and activation degree of MR in different tissues will significantly increase. Overactivation of MR is one of the important causes of adverse renal heart outcomes (Jaisser and Farman, 2016), among which the renin-angiotensin-aldosterone system (RAAS) pathway leads to over activation of MR, and non RAAS pathways caused by factors such as high salt and high sugar can also mediate over activation of MR. RAAS inhibitor (RAASI) is the standard treatment scheme for diabetes related CKD, but research has found that it has some limitations. Some patients are receiving RAASI treatment, whether angiotensin converting enzyme inhibitor (ACEI) or angiotensin receptor blocker (ARB), there is aldosterone escape phenomenon (Schwenk, Hirsch, and Bomback, 2015), which can not fully block the excessive activation of MR; And drugs that act on non RAAS pathways can only indirectly inhibit MR overactivation. Therefore, in clinical practice, there is a greater need for drugs that directly act on MR, namely, MRA. Some clinical trials have demonstrated that MRAs can reduce proteinuria and blood pressure, and when combined with renin-angiotensin system blockers, they can provide additional renal protection in patients with diabetic kidney disease (DKD) (Sato, Hayashi, and Saruta, 2005; Schjoedt et al., 2005; Schjoedt et al., 2006; Mehdi et al., 2009). In clinical practice, traditional MRA is a steroid drug, and its representative drugs spironolactone and eplerenone were approved by the US FDA in 1960 and 2002, respectively (Ménard, 2004; Barrera-Chimal et al., 2019a). Currently, randomized controlled trials of the steroidal MRAs spironolactone and eplerenone have provided robust evidence for the clinical use of MRAs in the treatment of heart failure (Pitt et al., 1999; Pitt et al., 2003; Zannad et al., 2011), while the protective effect of MRAs in cardiovascular disease may be translated into cardiovascular protection in patients with DKD (Barrera-Chimal et al., 2022). However, their steroid structure causes many adverse effects, such as hyperkalemia, male breast development, sexual dysfunction and so on (Lainscak et al., 2015). New nonsteroidal MRAs will increase the application of MRAs in HF patients, especially for patients complicated with advanced CKD and/or diabetes, and it is possible to further reduce their cardiovascular mortality (Pitt, Pedro Ferreira, and Zannad, 2017).

Currently, a variety of nonsteroidal MRAs have completed phase II and III clinical trials, including finerenone, esaxerenone, and apararenone. The indications for evaluation include hypertension, heart failure complicated with CKD and/or diabetes, and DKD (Capelli et al., 2020). In January 2019, the Pharmaceuticals and Medical Devices Agency (PMDA) in Japan approved the indication of esaxerenone for the treatment of hypertension. In July 2021, the US Food and Drug Administration (FDA) approved the indication of finerenone for reducing the progression of severe kidney disease and preventing the development of cardiac complications in patients with type 2 diabetes and CKD (Liu and Sheng-Qiang, 2022). In June 2022, finerenone was also marketed in China for adult patients with CKD associated with type 2 diabetes (eGFR ≥25 to <75 mL/min/1.73 m^2^ with albuminuria) to reduce the risk of sustained eGFR decline and end-stage renal disease. Given the relatively short development and marketing time of these drugs, this meta-analysis aims to evaluate the efficacy and safety of nonsteroidal MRAs in treating CKD.

## 2 Materials and methods

### 2.1 Search strategy

We searched PubMed, Embase, Cochrane Library, SinoMed, China National Knowledge Infrastructure (CNKI) and WanFang Med online from inception to 22 August 2023, with the search terms “Nonsteroidal Mineralocorticoid receptor antagonist” OR “Finerenone” OR “Kerendia” OR “BAY 94-8862” OR “Esaxerenone” OR “CS-3150” OR “Apararenone” OR “MT-3995” and “Renal Insufficiency, Chronic” OR “Diabetic nephropathy”. Supplementary Table S1 presents the detailed search strategy.

### 2.2 Inclusion and exclusion criteria

Studies meeting these criteria were considered eligible: (1) Type of study: RCT; (2) patients (age ≥18 years) with CKD (UACR ≥30 mg/g and eGFR ≤90 mL/min/1.73 m^2^ for more than 3 months); (3) oral nonsteroidal MRA as an intervention at the doses in the instructions or that referred to phase III clinical trials; (4) placebo or any other drugs applied in the control group; (5) at least one interested outcome was reported; (6) RCTs published in English or Chinese. The exclusion criteria were as follows: (1) meta-analysis, review, case report, conference, and letter; (2) animal experiments; (3) patients receiving renal replacement therapy; (4) single-arm, open-label study.

### 2.3 Data extraction

Two reviewers independently extracted data from the included studies, and any disagreements were resolved through consultation with a third reviewer to reach a consensus. The extracted data included the first author, publication time, country, intervention time, drug dose, number of participants, gender, outcomes and results. The outcomes included ① sustained decrease of 40% in the eGFR from baseline; ②the change from the baseline in eGFR; ③composite renal outcome: including renal failure, a sustained decrease in eGFR ≥40% compared to the baseline, or death from renal causes; ④the mean of UACR from baseline; ⑤ composite cardiovascular outcome: including death from cardiovascular causes, nonfatal myocardial infarction, nonfatal stroke, or hospitalization due to heart failure; ⑥hospitalization for heart failure; ⑦change in NT-proBNP; ⑧any adverse event; ⑨Hyperkalemia and blood K^+^level increased.

### 2.4 Quality assessment

Two investigators independently evaluated the risk of bias of the included studies and cross-checked the results. Risk of bias was explored according to the Cochrane Handbook for Systematic Reviews of Interventions (the detailed list was as follows: random sequence generation (selection bias), allocation concealment (selection bias), blinding of participants and personnel (performance bias), blinding of outcome assessment (detection bias), incomplete outcome (attrition bias), selective reporting (reporting bias), and other bias.

### 2.5 Statistical methods

Stata software version 17.0 was used to perform statistical analysis. We used weighted mean differences (WMDs) and their associated 95% confidence intervals (CIs) to assess continuous outcomes. Besides, we used risk ratios (RRs) and their associated 95% CIs to assess dichotomous outcomes. Statistical heterogeneity was assessed using the I^2^ test. If significant heterogeneity was not present (I^2^ < 50%, *p* ≥ 0.05), we used fixed effects models to pool outcomes; we used random effects models when significant heterogeneity was present (I^2^ ≥ 50%, *p* < 0.05). We preliminarily assessed the publication bias by funnel plot, and then the Egger test was used to do further analyses. Sensitivity analyses were performed by removing one study at a time to explore whether the heterogeneity was significantly reduced. The efficacy and safety of included drugs was considered significantly different if *p* < 0.05 and the 95% CI did not contain a WMD = 0 or an RR = 1.

## 3 Results

### 3.1 Study characteristics

We identified 1,602 articles from the electronic database, PubMed (309), Embase (603), Cochrane Library (112), Web of Science (535), CNKI (14), WanFang Med Online (8), SinoMed (21). After the removal of duplicate data (702), and records excluded due to topics and type of articles (811), 89 full-text articles were assessed for eligibility, of which 11 studies met the inclusion criteria (Pitt et al., 2013; Bakris et al., 2015; Filippatos et al., 2016; Sato et al., 2016; Katayama et al., 2017; Ito et al., 2019; Bakris et al., 2020; Ito et al., 2020; Bakris et al., 2021; Pitt et al., 2021; Wada et al., 2021). Figure 1 shows the literature screening process. A total of 15,817 patients were included in this meta-analysis. The characteristics of the included studies are presented in Supplementary Table S2.

**FIGURE 1:** Flow diagram of the screening process.

### 3.2 Evaluation of the risk of bias of selected studies

The risk of bias for the included RCTs was assessed using the Cochrane Risk-of-Bias tool. Five RCTs had an unclear risk of bias for blinding of participants and personnel (performance bias), four for blinding of outcome assessment (detection bias), and five for the imcomplete outcome data (attrition bias). The details regarding the risk of bias in each study are presented in Figure 2.

**FIGURE 2:** **(A)** Risk of bias graph **(B)** Risk of bias summary.

### 3.3 Results of the meta-analysis

#### 3.3.1 Sustained decrease of ≥40% in eGFR from baseline

Four RCTs reported (n = 13,500) the incidence of a sustained decrease of 40% in the eGFR from baseline between the nonsteroidal MRA group and placebo group. No significant heterogeneity was observed in the study (I^2^ = 0%, *p* = 0.642) (Figure 3A). Using the fixed effects model, the results suggested that after nonsteroidal MRA treatment, the proportion of patients with a decrease in eGFR of ≥40% from the baseline was significantly lower than that of placebo [RR = 0.85, 95% CI (0.78, 0.92), *p < 0.001*]. In addition, two RCTs (n = 673) reported the incidence of a sustained decrease of 40% in the eGFR from baseline between the nonsteroidal MRA and eplerenone, and no significant difference was observed (I^2^ = 14.0%, *p* = 0.281) (Figure 3B). Using the fixed effects model, the results suggested that the nonsteroidal MRA group and the eplerenone group had no significant difference [RR = 0.57, 95% CI (0.18, 1.79), *p = 0.335*].

**FIGURE 3:** **(A)** Meta-analysis results of sustained ≥40% decrease in eGFR from baseline in Nonsteroidal MRA vs. Placebo. **(B)** Meta-analysis results of sustained ≥40% decrease in eGFR from baseline in Nonsteroidal MRA vs. Eplerenone.

#### 3.3.2 The change from the baseline level in eGFR

Five RCTs (n = 6,609) reported the change from the baseline in eGFR. The results did not have significant heterogeneity (I^2^ = 36.8%, *p* = 0.176) (Figure 4). The difference was statistically significant [WMD = −2.83, 95% CI (−3.95, −1.72), *p < 0.001*], indicating that the eGFR in the nonsteroidal MRA group was lower than that in the placebo group.

**FIGURE 4:** Meta-analysis results of changes in the eGFR from the baseline for Nonsteroidal MRA vs. placebo.

#### 3.3.3 Composite renal outcome

Three RCTs (n = 13,652) reported the composite renal outcome, including renal failure, a sustained decrease in eGFR of ≥40% compared to the baseline, or death from renal causes. No significant heterogeneity was found in the study (I^2^ = 0.0%, *p = 0.642*) (Figure 5). Using the fixed effects model, the results showed that the composite renal outcome of patients after nonsteroidal MRA treatment was significantly lower than that of placebo [RR = 0.86, 95% CI (0.79, 0.93), *p < 0.001*].

**FIGURE 5:** Meta-analysis results of the effect of Nonsteroidal MRA vs. Placebo on composite kidney outcome.

#### 3.3.4 Mean of the UACR from baseline

Eight trials compared the mean of UACR from baseline between nonsteroidal MRA (n = 7,296) and placebo (n = 6,727) groups of CKD patients. The results showed significant heterogeneity (I^2^ = 85.7%, *p < 0.001*) (Figure 6). Using the random effects model, the mean of UACR from baseline was significantly lower for nonsteroidal MRA than for placebo [WMD = −0.41, 95% CI (−0.49, −0.32), *p < 0.001*], indicating that nonsteroidal MRA can effectively reduce UACR.

**FIGURE 6:** Meta-analysis results of mean of the UACR from the baseline for Nonsteroidal MRA vs. Placebo.

#### 3.3.5 Composite cardiovascular outcome

Four studies (n = 13,658) reported the composite cardiovascular outcome between nonsteroidal MRA group and placebo group, including death from cardiovascular causes, nonfatal myocardial infarction, nonfatal stroke, or hospitalization due to heart failure. No significant heterogeneity was found among the studies (I^2^ = 0.0%, *p* = 0.845) (Figure 7). Using the fixed effects model, the incidence of cardiovascular events in the nonsteroidal MRA group was significantly lower than that in the placebo group [RR = 0.88, 95% CI (0.80, 0.95), *p* = 0.003].

**FIGURE 7:** Meta-analysis results of the effect of Nonsteroidal MRA vs. Placebo on composite cardiovascular outcome.

#### 3.3.6 Hospitalization for heart failure

Two studies (n = 13,026) reported the number of hospitalization for heart failure between nonsteroidal MRA group and placebo group. No significant heterogeneity was found among the studies (I^2^ = 23.1%, *p* = 0.254) (Figure 8). Using the fixed effects model, the incidence of hospitalization for heart failure in the nonsteroidal MRA group was significantly lower than that in the placebo group [RR = 0.79, 95% CI (0.67, 0.92), *p* = 0.003].

**FIGURE 8:** Meta-analysis results of the effect of Nonsteroidal MRA vs. Placebo on hospitalization for heart failure.

#### 3.3.7 Change in NT-proBNP

Two RCTs reported change in NT-proBNP between the nonsteroidal MRA group and eplerenone group. Three results were included in the analysis: ①median change from baseline in NT-proBNP concentration [WMD = −278.89, 95% CI (−638.03, 80.24), *p = 0.128*], ②the proportion of patients who had an NT-proBNP level decrease of 30% compared with baseline was similar in the finerenone group and the eplerenone group [RR = 1.03, 95% CI (0.84,1.25), *p* = 0.786], ③ratio of NT-proBNP at day 90 to baseline [WMD = 0.05, 95% CI (−0.42,0.51), *p = 0.848*]. Change in NT-proBNP between the two groups had no significant difference (Figure 9).

**FIGURE 9:** **(A)** Meta-analysis results of Nonsteroidal MRA vs. Eplerenone on median change from baseline in NT-proBNP concentration **(B)** Meta-analysis results of Nonsteroidal MRA vs. Eplerenone on treatment comparison for proportion of patients with a relative decrease in NT-proBNP of >30% from vaseline **(C)** Meta-analysis results of.

#### 3.3.8 Any adverse event

Eight RCTs (n = 14,511) reported any adverse event. No significant heterogeneity was found (I^2^ = 0.0%, *p* = 0.599) (Figure 10A). Using the fixed effects model, there was no significant difference between the nonsteroidal MRA group and the placebo group [RR = 1.00, 95% CI (0.99, 1.01), *p* = 0.909].

**FIGURE 10:** **(A)** Meta-analysis results of any adverse events in Nonsteroidal MRA vs. placebo **(B)** Meta-analysis results of any adverse events in Nonsteroidal MRA vs. Eplerenone.

In the comparison with the eplerenone group, 2 RCTs (n = 942) were enrolled, and the results had significant heterogeneity (I^2^ = 53.1%, *p* = 0.144) (Figure 10B). Using the random effects model, no significant difference was observed in the incidence of any adverse events between the nonsteroidal MRA group and the eplerenone group [RR = 0.89, 95% CI (0.77, 1.02), *p* = 0.101].

#### 3.3.9 Hyperkalemia and blood K^+^ level increased

Eight RCTs (n = 14,607) reported the incidence of hyperkalemia or serum potassium ≥5.6 or ≥6.0 mmol/L. The results suggested that the heterogeneity was small (I^2^ = 0.0%, *p* = 0.743) (Figure 11A). Using the fixed effects model, the incidence of hyperkalemia in the nonsteroidal MRA group was higher than that in the placebo group [RR = 2.05, 95% CI (1.85, 2.28), *p* < 0.001].

**FIGURE 11:** **(A)** Meta-analysis results of Hyperkalemia in Nonsteroidal MRA vs. Placebo. **(B)** Meta-analysis results of Hyperkalemia in Nonsteroidal MRA vs. Eplerenone **(C)** Meta-analysis results of blood K + level increased in Nonsteroidal MRA vs. Placebo.

In the comparison with eplerenone group, 2 RCTs (n = 917) were enrolled, and the results had no significant heterogeneity (I^2^ = 0.0%, *p* = 0.757) (Figure 11B). The fixed model showed no significant difference in hyperkalemia between the nonsteroidal MRA group and eplerenone group [RR = 0.95, 95%CI (0.48, 1.88), *p* = 0.875].

In addition, four trials (n = 1,302) also reported the incidence of blood K^+^ level increased. The studies did not show significant heterogeneity (I^2^ = 0.0%, *p* = 0.902) (Figure 11C). The results showed that the incidence of blood K^+^ level increased in the nonsteroidal MRA group was higher than the placebo group by using a fixed effect model [RR = 5.21, 95%CI (2.57, 10.56), *p* < 0.001].

### 3.4 Sensitivity analysis

Sensitivity analysis using the mean of UACR from baseline as an indicator. The results showed that there was no statistically significant difference between the overall effective rate after each study was excluded and that before it was excluded (*p* > 0.05), indicating that the results in this study are stable (Figure 12A).

**FIGURE 12:** **(A)** Decreased level of UACR in patients compared to the baseline sensitivity analysis **(B)** Funnel plot of the decrease in UACR for patients compared to the baseline **(C)** Egger’s test.

### 3.5 Publication bias analysis

The funnel plot was drawn using the mean of UACR from baseline as an indicator. The plot could not accurately determine the results. Therefore, an Egger test was performed, and the *p*-value of Egger’s test was 0.150, indicating that there was a low possibility of publication bias in the present study (Figures 12B, C).

## 4 Discussion

Kidney diseases have a profound impact on global health, not only increasing morbidity and mortality globally but also serving as a key risk factor for cardiovascular diseases. CKD is preventable and treatable, and should be a priority for global health policy decision-making (Collaboration, GDB Chronic Kidney Disease, 2020).

In mammals, aldosterone is the main mineralocorticoid (Rossier, Baker, and Studer, 2015). Aldosterone has been associated with inflammation, fibrosis, vascular injury, and end-organ failure since its discovery (Ferreira et al., 2021). In an inactive state, MR binds to chaperones such as HSP90 and KFBP52 in the cytoplasm. In the presence of aldosterone, MR dissociates from chaperones and binds to aldosterone, entering the nucleus. By binding to the hormone response element (HRE) in DNA, it aggregates co transcription factors and expresses genes related to inflammation and fibrosis, leading to an increase in inflammation and fibrosis in the heart and kidney tissues (Yang and Fuller, 2012; Brown, 2013). There is a growing body of evidence that MR is also expressed in vascular endothelial cells and vascular smooth muscle cells podocytes, mesangial cells, and renal fibroblasts, cardiomyocytes, coronary endothelial and inflammatory cells, such as macrophages (Bauersachs, Jaisser, and Toto, 2015). Besides the kidney, there are numerous other cells and organs that express theMR, including the heart, eyes, and skin. In these tissues, activation of MR mediates pathological changes. After direct binding of MRAs and MR, their conformation is altered, directly inhibiting the expression of inflammation related genes (Jaisser and Farman, 2016; Epstein, 2021).

Preclinical data suggests that MR antagonism has the potential to treat or delay kidney disease due to various etiologies, including ischemic kidney disease, diabetic and hypertensive nephropathy, glomerulonephritis, and calcineurin inhibitor toxicity in the context of kidney transplantation (Barrera-Chimal et al., 2019b). Inflammation is the main trigger of renal fibrosis. MRAs directly regulate the inflammatory cell function in kidneys, induce suppression of proinflammatory cytokines, chemoattractants, and pro-oxidants, and increase anti-inflammatory cytokines in renal tissue (Patel et al., 2020). Thus, MRAs can inhibit renal fibrosis and protect the kidney. Chronic kidney lesions can be observed in animal models of ischemia or drug-induced acute kidney injury (AKI) after a few weeks (Wei et al., 2019). Recent epidemiological studies have shown that AKI significantly increases the risk of developing CKD and end-stage renal disease (ESRD) in the future. The evidence from clinical studies, meta-analyses, and animal models strongly supports the notion that AKI is closely associated with the development of CKD (Zhu et al., 2022). A large number of preclinical studies have now shown that MRA can prevent the transformation of AKI to CKD, playing a role in kidney protection (Barrera-Chimal et al., 2015; Lattenist et al., 2017; Barrera-Chimal et al., 2019a).

Although nonsteroidal MRA and steroidal MRA bind to the same MR ligand-binding domain, there are some differences in molecular action mechanisms. Spironolactone and eplerenone are passive MR antagonists that can rapidly dissociate from the receptors. Automatic quantification of the subcellular distribution of MR demonstrated that finerenone, a nonsteroidal MRA, more effectively delays aldosterone-induced nuclear accumulation of MR compared to spironolactone. Unlike spironolactone, finerenone inhibits MR, steroid receptor coactivator-1, and RNA polymerase II binding at the regulatory sequence of the SCNN1A gene. It also significantly reduces basal MR and steroid receptor coactivator-1 recruitment, revealing a specific and previously unrecognized inactivating mechanism on MR signaling. The highly potent and selective MR antagonist finerenone specifically impairs several critical steps of the MR signaling pathway and represents a promising new generation MRA (Amazit et al., 2015). Esaxerenone, another nonsteroidal MRA, also binds to the MR ligand-binding domain (MR-LBD) in a unique manner with large side-chain rearrangements, distinct from those of previously published MR antagonists (Takahashi et al., 2020) Moreover, nonsteroidal MRAs have a lower risk of hyperkalemia than steroidal MRAs (Barrera-Chimal et al., 2022). Therefore, nonsteroidal MRA is mechanistically different from steroidal MRA, and its novelty, unique potency and selectivity mean that they may be a promising new generation of MR antagonists.

This study compared the efficacy and safety of nonsteroidal MRAs (including finerenone, esaxerenone, apararenone, and KBP-5074) in patients with CKD. The results showed that, compared to placebo, nonsteroidal MRAs could effectively reduce the proportion of patients experiencing a ≥40% decrease in eGFR, the mean urine albumin-to-creatinine ratio (UACR) from baseline, hospitalization for heart failure, and the composite renal and cardiovascular outcomes. It is suggested that nonsteroidal MRAs have a protective effect on the hearts and kidneys of patients with CKD. Our inclusion criteria were CKD, with or without diabetes. However, from the perspective of the included RCTS, most of the studies involved CKD with diabetes, and only four RCTs (Pitt et al., 2013; Filippatos et al., 2016; Sato et al., 2016; Bakris et al., 2021) included CKD without diabetes. Since the number of patients without diabetes is limited, the efficacy and safety of non-steroidal MRAs in patients without diabetes remain unclear. Therefore, further RCTs with larger sample sizes are required to provide more conclusive evidence.

eGFR is an important indicator of renal function evaluation. In this meta-analysis, the eGFR in the nonsteroidal MRA group was slightly lower than that in the placebo group compared to the baseline level. This may be related to the short duration of the study, as the follow-up data at the 4 months was selected for this meta-analysis. However, it is noteworthy that from 32 months onwards, the eGFR of the finerenone group was higher than that of the placebo group from baseline until the end of the 44-month observation period (Bakris et al., 2020). Moreover, another study showed that eGFR decreased during the early stage of treatment, but gradually recovered to the baseline level after treatment (Ito et al., 2019). It suggests that the impact of nonsteroidal MRA on eGFR levels may vary over time, necessitating regular monitoring of kidney function and longer clinical trial observation.

In a patient population with multiple comorbidities and advanced CKD, where almost 55% of the patients had a baseline eGFR of <45 mL per minute per 1.73 m^2^, and were at high risk for kidney and cardiovascular events, the benefits of finerenone were observed after 12 months for the kidney outcome and as early as 1 month for the cardiovascular outcome. These benefits persisted throughout the trial (Bakris et al., 2020). Similarly, the present study suggested that in comparing the incidence of the composite cardiovascular outcome (such as death from cardiovascular causes, nonfatal myocardial infarction, nonfatal stroke, or hospitalization for heart failure), the incidence rate of the nonsteroidal MRA group was significantly reduced.

In terms of safety, no significant difference was observed in the incidence of any adverse events between the nonsteroidal MRA group and the placebo group, indicating that the safety was well, but the main adverse reaction requiring attention was hyperkalemia. The ARTS trial using spironolactone as a control (Pitt et al., 2013) showed that the incidence of hyperkalemia using finerenone 10 mg/d was lower than that of taking spironolactone 25–50 mg/d (4.5% and 11.1%), but the maximum dose of finerenone is 20 mg/d in package insert, which is higher than it in the ARTS trial.

Although the risk of hyperkalemia in nonsteroidal MRA group was lower than that in spironolactone group, it was higher than the placebo group [RR = 2.05, 95% CI (1.85, 2.28), *p* < 0.001]. Therefore, the risk of increased serum potassium still needs to be vigilant. It is necessary to monitor serum potassium during treatment. In the management of chronic diseases, dietary management should be strengthened to limit the intake of high-potassium foods or the use of potassium-lowering drugs when necessary. In recent years, treatment with some new types of potassium ion adhesives significantly reduced serum K+ and maintained normokalemia in hyperkalemic patients with CKD (Weir et al., 2018).

In addition to the comparison with placebo, this meta-analysis also compared nonsteroidal MRA and eplerenone. Some studies have shown that spironolactone is approximately 40-fold more potent than eplerenone in blocking aldosterone activation of MR. However, eplerenone exhibits significantly greater selectivity than spironolactone at androgen, progesterone, and glucocorticoid receptors (Garthwaite and McMahon, 2004). The EPHESUS trial, which studied more than 6,600 post-acute myocardial infarction (AMI) patients, demonstrated that the addition of eplerenone to optimal medical therapy reduced morbidity and mortality among patients with AMI complicated by left ventricular dysfunction and heart failure (Pitt, Remme, Zannad, Neaton, Martinez, Roniker, Bittman, Hurley, Kleiman, and Gatlin, 2003). Approval of eplerenone for treatment of heart failure post-AMI in the US was received in October 2003 (Garthwaite and McMahon, 2004).

In this meta-analysis, we also compared nonsteroidal MRA to eplerenone, this is something that has rarely been covered in previous meta-analyses. No significant difference was observed in any adverse events or the incidence of hyperkalemia, suggesting that nonsteroidal MRA may have a similar safety profile as eplerenone. There was no significant difference in the proportion of patients with a decrease in eGFR of ≥40% from the baseline, suggesting that the advantage of nonsteroidal MRA in kidney protection is not significant. The change of NT-proBNP level was similar in the finerenone and eplerenone groups too. However, ARTS-HF compared with patients in the eplerenone group, patients in the finerenone 10-20 mg dose group had the greatest reduction in the composite outcome including death from any cause, cardiovascular hospitalization, or emergency presentation to hospital, compared with patients in the eplerenone group (HR: 0.56; 95% CI: 0.35, 0.90) (Filippatos et al., 2016). Preclinical studies have also shown that finerenone potently prevents cardiac fibrosis and improves strain parameters. Isoproterenol-induced cardiac fibrosis and macrophage invasion were potently blocked by finerenone, whereas eplerenone had no significant effect. Speckle tracking echocardiography revealed a significant improvement of global longitudinal peak strain by finerenone, an effect less prominent with eplerenone (Grune et al., 2018). This suggests that finerenone may be superior in cardiovascular aspects, but more clinical trials are needed for confirmation.

A preclinical study has shown that the combination of finerenone, a nonsteroidal MRA, and empagliflozin, a sodium-glucose co-transporter 2 (SGLT2) inhibitor, confers cardiovascular protection in preclinical models of hypertension-induced cardiorenal disease. When administered at low dosages, the combination of these two independent modes of action effectively reduced important functional parameters such as proteinuria and blood pressure, plasma markers including creatinine and uric acid, and cardiac and renal lesions as determined by histopathology. This reduction in mortality further highlights the strong potential for combined clinical use in cardiorenal patient populations (Kolkhof et al., 2021a). The addition of the nonsteroidal MRA finerenone to optimal renin-angiotensin system (RAS) blockade resulted in reduced cardiovascular (CV) and kidney outcomes in patients with CKD and type 2 diabetes (T2D). Furthermore, hyperkalemia-related discontinuation was low and manageable. Therefore, the use of the nonsteroidal MRA finerenone has the potential to target the important downstream portion of the RAAS cascade, either as a monotherapy or in combination with a sodium-glucose co-transporter 2 inhibitor (SGLT2i), among a broad population of patients with cardiovascular and renal diseases (Kolkhof et al., 2021b). MRAs increase the serum potassium concentration and the risk of hyperkalemia, but in contrast, SGLT2 inhibitors may reduce the risk of hyperkalemia (Provenzano et al., 2022). The study of Neuen B.L included 6 RCTs with 49,875 participants, and the conclusion was that SGLT2 inhibitors reduce the risk of serious hyperkalemia in people with type 2 diabetes at high cardiovascular risk and/or with CKD, without increasing the risk of hypokalemia (Neuen et al., 2022). Therefore, the combined use of SGLT2 inhibitors or RAS blockade may bring greater benefits to CKD patients, but more high-quality clinical trials are needed to support this hypothesis.

This study also had several limitations. First, most of the RCTs were compared with the placebo group, and only two were compared with eplerenone. More comparisons with other active drugs, such as ACE inhibitors/angiotensin receptor blockers (ARBs) and sodium-glucose cotransporter-2 (SGLT-2) inhibitors, which have clear evidence of cardio-renal protection, are needed to further evaluate the efficacy and safety of nonsteroidal MRAs. Second, the included studies comprised only published literature, excluding conference reports and other related research findings. The limited number of studies, all of which were phase II or III clinical trials sponsored by the company, may introduce publication bias. Third, only two trials had a long duration, while most other trials were of short duration, making it difficult to clearly assess the long-term effects of nonsteroidal MRAs on patients with CKD. More long-term, large-scale, multicenter clinical studies after drug marketing are warranted to obtain more rigorous and reliable clinical evidence.

## 5 Conclusion

Nonsteroidal MRAs can reduce the incidence of end-stage renal disease and cardiovascular adverse events in patients. Although there was still a risk of hyperkalemia compared to placebo, there was no significant difference in any adverse events compared to either placebo or eplerenone. It has become a new option for drug treatment of CKD patients, but more clinical trials are still needed to verify its efficacy and safety. Especially further direct comparison of the non-steroidal MRAs to eplerenone in view of the relatively small number of patients reviewed are needed.

## Data Availability

The original contributions presented in the study are included in the article/Supplementary Material, further inquiries can be directed to the corresponding author.
